The article "The Identified Hub Gene GlcN in Osteoarthritis Progression and Treatment" was published in 2021. Journal: Comput Math Methods Med.

# The Identified Hub Gene GlcN in Osteoarthritis Progression and Treatment

**DOI:** 10.1155/2021/5499450

**Published:** 2021-10-31

**Authors:** Jingsheng Liu, Xiaoli Dong, Yining Liu, Kai Wang, Shuanhu Lei, Mingxuan Yang, Haiyuan Yue, Haijun Feng, Kai Feng, Kang Li, Jianwei Zhou, Yanqiang Chen, Wenjia Du, Xuewen Kang, Yayi Xia

**Affiliations:** ^1^The Fourth Ward of Orthopedics Department of the Second Hospital of Lanzhou University, No. 80 Cuiyingmen, Lanzhou City, Gansu Province 730000, China; ^2^Department of Physiology, Gansu University of Traditional Chinese Medicine, Chengguan District, Lanzhou City, Gansu Province 730030, China; ^3^T.C Jasper School, Plano Independent School District, 6800 Archgate Dr. Plano, TX 75024, USA

## Abstract

**Background:**

As a chronic disease, osteoarthritis has caused great trouble to the health of middle-aged and elderly people. Studies have shown that glucosamine (GlcN) can be used to abate the progression and improve this disease. Based on this point of view, we try to verify the connection between GlcN and osteoarthritis and find more effective biomarkers.

**Methods:**

We downloaded the GSE72575 data set from the GEO database, and used the R language to perform DEG analysis on the gene expression profile of the samples. Next, the GO function and the KEGG signaling pathways were analyzed through the DAVID database, and then, the KEGG pathways enriched in the gene set were analyzed based on GSEA. Then, the PPI network of DEGs was constructed based on the STRING online database, and finally, the hub genes were selected by Cytoscape.

**Results:**

Three GlcN-treated MH7A cell treatment groups and 3 control groups in the GSE72575 data set were studied. Through analysis, there were 52 DEGs in these samples. Then, through GO, KEGG, and GSEA, regulation of endoplasmic reticulum stress-induced intrinsic apoptotic signaling pathway, FoxO signaling pathway, JAK-STAT signaling pathway, PI3K-Akt signaling pathway, TGF-beta signaling pathway, and ECM receptor interaction were involved in the regulatory mechanisms of the osteoarthritis pathogenesis. After that, the hub genes IL6 and DDIT3 were identified through PPI network construction and analysis. And it was found that IL6 was lowly expressed in the group with GlcN-treated MH7A cells, while DDIT3 was highly expressed.

**Conclusion:**

The above results provide a basis for GlcN to participate in the treatment of osteoarthritis and a possibility for finding effective therapeutic targets.

## 1. Background

Osteoarthritis is a progressive chronic disease, also known as degenerative arthritis, senile arthritis, and hypertrophic arthritis [1]. As for the types of disease, it can be divided into primary osteoarthritis and secondary osteoarthritis [2]. The former is more common in middle-aged and elderly people, mainly manifesting as joint pain, stiffness, swelling, deformity, and so on due to articular cartilage damage. The latter is osteoarthritis lesions based on the original lesions and can occur in young adults. According to statistics, 80% to 90% of the 70-year-old population suffers from various degrees of osteoarthritis, and the incidence far exceeds that of cardiovascular disease [3]. At present, the etiology and specific pathogenesis of osteoarthritis are not clear, but it is acknowledged that there is a certain relationship with age, weight, genetics, occupation, etc. [4]. Clinically, it is usually to reduce the weight of the joints and to inhibit the process of the disease by excessive and large movements [5]. The early stage can be treated with drugs, and the later stage mainly relies on surgery for treatment. Most patients can recover after targeted treatment, but the prognosis of a few patients is not optimistic. Current studies have proved that glucosamine is effective in the treatment of osteoarthritis, and long-term use can relieve symptoms and improve body function [6]. Therefore, it is very important to determine the molecular biomarkers of osteoarthritis and the underlying molecular mechanisms of glucosamine to regulate osteoarthritis.

The article "The Identified Hub Gene GlcN in Osteoarthritis Progression and Treatment" was published in 2021. Journal: Comput Math Methods Med.

Glucosamine (GlcN) is natural amino monosaccharide necessary for the synthesis of proteoglycans in the matrix of human articular cartilage [7]. They are widely present in nature and can also be synthesized by the human body. GlcN can be used to repair articular cartilage, promote joint synovial fluid, and effectively reduce the friction of the joint surface [8]. It can also play an anti-inflammatory effect, reduce joint pain, improve joint function, and effectively prevent the development of osteoarthritis [9].

Microarray, also known as oligonucleotide array, is the product of the gradual implementation of the Human Genome Project and the rapid development and application of molecular biology [10]. The integration of microelectronics, life sciences, computer science, and photoelectrochemistry is one of the main technologies of the genome revolution. Microarray analysis can quickly identify all genes expressed at any time point and is suitable for screening differentially expressed genes (DEGs) [11]. It is of great significance for humans to explore the mysteries of life and reveal the nature of diseases and the realization of the Human Genome Project.

We applied microarray analysis to this study and identified DEGs through R language. Then, the Gene Ontology (GO) function and Kyoto Encyclopedia of Genes and Genomes (KEGG) pathway enrichment analysis of DEGs was performed using the Database for Annotation, Visualization and Integrated Discovery (DAVID). Next, based on gene set enrichment analysis (GSEA), the enriched KEGG gene set in the GlcN-treated MH7A cell group was analyzed. After that, the Search Tool for the Retrieval of Interacting Genes (STRING) database was used to construct a Protein-Protein Interaction (PPI) network to identify the hub genes. The above methods were used to verify the role of GlcN in osteoarthritis treatment and find relevant and effective biomarkers.

The article "The Identified Hub Gene GlcN in Osteoarthritis Progression and Treatment" was published in 2021. Journal: Comput Math Methods Med.

## 2. Materials and Methods

### 2.1. Microarray Data

We downloaded the GSE72575 gene expression data set from the Gene Expression Omnibus (GEO) data set (https://www.ncbi.nlm.nih.gov/geo/) and saved it in the form of series matrix files [12]. Three GlcN-treated MH7A cell treatment groups and 3 MH7A cell control groups were used in this study.

### 2.2. Data Preprocessing and DEG Screening

The data in GSE72575 were preprocessed, and probe annotations were carried out through R language. *P* < 0.05 was used as the screening condition for DEGs, and the final results were expressed in the form of heat maps.

### 2.3. GO Function and KEGG Pathway Enrichment Analysis

GO function analysis was used to study the function of the large-scale genome or transcriptome data, including biological process (BP), cellular component (CC), and molecular function (MF). Among them, BP was used to explain the biological processes that genes were involved in, CC was used to explain where the genes exist, and MF was used to explain the functions of genes at the molecular level. KEGG was an annotation of the function of the gene itself and analyzed the various pathways that the gene participated in. DAVID (http://david.ncifcrf.gov/) was a database for systematic and comprehensive analysis of large gene lists [13]. In this study, DAVID was used to analyze the functions of DEGs in GO and KEGG pathways. When *P* < 0.05, it was considered to be statistically significant.

### 2.4. GSEA

GSEA (https://www.gsea-msigdb.org/gsea/index.jsp) used a predefined gene set to sort genes according to the degree of differential expression in the two types of samples and then checked whether the predefined gene set was enriched at the top or bottom of the sorting table. In this study, GSEA was used to identify the enriched KEGG gene set in the GlcN-treated MH7A cell group.

### 2.5. PPI Network of DEGs

The STRING database (https://string-db.org/) was usually used to integrate the relationships between various proteins. We used this database to construct a PPI network diagram of DEGs and selected the hub genes we needed from the network diagram using Cytoscape. Genes with degree ≥ 4 were defined as hub genes.

The article "The Identified Hub Gene GlcN in Osteoarthritis Progression and Treatment" was published in 2021. Journal: Comput Math Methods Med.

## 3. Results

### 3.1. DEG Data Analysis

After analyzing the sample information in the GlcN-treated MH7A cell treatment groups and MH7A cell control groups in the GSE72575 data set, a total of 52 DEGs were identified, including 26 upregulated genes and 26 downregulated genes. The top 10 most significant DEGs were DIO2, SPX, GABRG1, SNORD54, MIR21, IL20RB, ASNS, GPR1, RNVU1-15, and BMP5, respectively.  Figure 1 showed the expression distribution of these DEGs in the two sets of samples.

### 3.2. GO Function and KEGG Pathway Enrichment Analysis

After analyzing the GO function and KEGG pathway enriched by DEGs through the DAVID database, we showed the results in Figures 2(a) and 2(b). For GO analysis, DEGs were mainly enriched in PERK-mediated unfolded protein response, long-chain fatty acid import, regulation of cell proliferation, positive regulation of STAT cascade, etc. in BP and only in GABA-A receptor complex in CC. In MF, DEGs were enriched in aminoacyl-tRNA ligase activity, cytokine receptor binding, cytokine activity, etc. In the KEGG signaling pathway, we analyzed that DEGs were significantly enriched in cytokine-cytokine receptor interaction, aminoacyl-tRNA biosynthesis, hematopoietic cell lineage, FoxO, JAK-STAT, PI3K-Akt, TGF-beta signaling pathway, and AGE-RAGE signaling pathway in diabetic complications.

### 3.3. GSEA

Figure 3 shows the enriched KEGG results of GSEA, in which the red part was the core gene set with higher expression. It could be seen from Figures 3(a)–3(f) that the genes of the GlcN-treated MH7A samples were enriched in 6 regulatory pathways, namely, ECM receptor interaction, complement and coagulation cascades, proteasome, spliceosome, focal adhesion, and Nod-like receptor signaling pathway.

### 3.4. PPI Analysis

The PPI network diagram of DEGs is shown in Figure 4 which contained 19 nodes and 17 edges. The yellow nodes, namely, IL6 and DDIT3, were the two hub genes identified which had a high correlation with other genes, and the next step was to analyze and study these two genes. It could be seen from the boxplot of Figure 5 that the expressions of the two hub genes were different in the treatment group and the control group. Among them, the expression level of IL6 in the treatment group of GlcN-treated MH7A cells was significantly lower than that in the control group of MH7A cells. On the contrary, the expression level of DDIT3 in the GlcN-treated MH7A samples was significantly higher than that in the control group.

## 4. Discussion

Osteoarthritis is a chronic disease that often occurs in the elderly [14]. In severe cases, it can cause complications, such as muscle atrophy and joint deformities [15]. For patients with osteoarthritis in the early stage, the disease can be relieved by taking anti-inflammatory and analgesic drugs [16]. In the later stage, only drug treatment cannot achieve the desired therapeutic effect. If necessary, surgical treatment is still required [17]. But at present, we only know that genetics, obesity, inflammation, trauma, and other factors can cause diseases, and the specific pathogenesis is still unclear [18]. Previous studies have shown that GlcN is often used in the treatment of patients with osteoarthritis [19]. Therefore, the main purpose of this study is to verify the relationship between GlcN and osteoarthritis and to find effective biomarkers for osteoarthritis.

The article "The Identified Hub Gene GlcN in Osteoarthritis Progression and Treatment" was published in 2021. Journal: Comput Math Methods Med.

The background of this study was based on the GSE72575 data set. We chose 3 GlcN-treated MH7A cell treatment groups and 3 MH7A cell control groups. After analyzing the information in the sample through R language, 52 DEGs were obtained. Later, we analyzed the enrichment of these DEGs in GO and KEGG using the DAVID database and found that in GO term, these DEGs were significantly enriched in PERK-mediated unfolded protein response, long-chain fatty acid import, regulation of endoplasmic reticulum stress-induced intrinsic apoptotic signaling pathway, GABA-A receptor complex, aminoacyl-tRNA ligase activity, cytokine receptor binding, anion channel activity, etc. The study by Hosseinzadeh et al. mentions that active oxygen destroys cartilage homeostasis through oxidative stress, induces cell death, and promotes catabolism. This process is the main cause of osteoarthritis. Then, it is seen that the apoptosis signal pathway is involved in the bone the biological process of arthritis [20]. In the KEGG signaling pathway, we analyzed that DEGs were significantly enriched in FoxO, JAK-STAT, PI3K-Akt, and TGF-beta signaling pathways, etc. The study by Ma et al. analyzed the regulatory role of the FoxO signaling pathway in bone cell function and confirmed that FoxO dysfunction in bone cells would cause osteoarthritis, osteoporosis, and other bone diseases [21]. Malemud and Pearlman believe that the increase in the level of inflammatory cytokines is one of the reasons leading to the progress of rheumatoid arthritis and bone and joint talk. Research has found that inflammatory cytokines activate a variety of signal pathways, including the JAK/STAT signal pathway. Therefore, it is confirmed that this signaling pathway is involved in the occurrence and progression of osteoarthritis [22]. Sun et al. take the role of the PI3K/AKT/mTOR signaling pathway in osteoarthritis as the research goal and discussed and summarized the role of this signaling pathway in disease development and treatment [23]. Not only that, Fang et al. also discussed and analyzed the role of the TGF-beta 1 signaling pathway in the occurrence and development of osteoarthritis and believed that this signaling pathway has a “conflict” phenomenon with the occurrence of osteoarthritis [24].

The article "The Identified Hub Gene GlcN in Osteoarthritis Progression and Treatment" was published in 2021. Journal: Comput Math Methods Med.

Then, we analyzed the enriched KEGG gene sets in the GlcN-treated MH7A samples according to GSEA and found that these genes were related to ECM receptor interaction, complement and coagulation cascades, proteasome, spliceosome, focal adhesion, and Nod-like receptor signaling pathway. Theocharis et al. introduce the role and pathways of ECM in osteoarthritis, fibrosis, cancer and genetic diseases, and other diseases, so it can prove that there is a certain connection between ECM receptor interaction and osteoarthritis [25]. Mianehsaz et al. find in the study the role of bone marrow mesenchymal stem cell-derived exons in the treatment of osteoarthritis, cartilage destruction, and loss of extracellular matrix which are important factors in affecting the occurrence of osteoarthritis [26].

After that, the PPI network diagram of DEGs was constructed from the STRING database, and two hub genes were identified, namely, IL6 and DDIT3. The expression levels of these two genes in the two sets of samples were analyzed afterwards, and the results showed that IL6 expression was higher in the MH7A cell control group, while DDIT3 expression was higher in the GlcN-treated MH7A cell group. DDIT3 participates in adipogenesis and erythropoiesis, is activated by endoplasmic reticulum stress, and promotes cell apoptosis [27]. This gene was fused with chromosome 16 FUS or chromosome 22 EWSR 1 to produce a chimeric protein in myxoid liposarcoma or Ewing's sarcoma [28]. It is usually expressed in myxoid liposarcoma and liposarcoma [29]. Although there was no research to prove the efficacy of these two genes in the pathogenesis of osteoarthritis, our research has shown that IL6 and DDIT3 can act as downregulated genes and upregulated genes in GlcN-treated cells, respectively. GlcN might have a special role in osteoarthritis progression by regulating the expression of these two genes. This study still has limitations. First, the expression profile of DEGs needs to be verified by clinical samples. Secondly, a further experimental study is required to confirm the function of the hub genes in osteoarthritis.

In short, after analyzing the two sets of samples in the GSE72575 data set, a total of 52 DEGs were identified. ECM receptor interaction and signaling pathways including endoplasmic reticulum stress-induced intrinsic apoptotic, FoxO, JAK-STAT, PI3K-Akt, and TGF-beta were all related to the pathogenesis of osteoarthritis through enrichment analysis. Finally, we identified two hub genes, IL6 and DDIT3, and found that IL6 was low-expressed in MH7A cells treated with GlcN, while DDIT3 was highly expressed. The above results verified that GlcN was involved in the treatment of osteoarthritis and provided the possibility to find effective biomarkers for osteoarthritis.

The article "The Identified Hub Gene GlcN in Osteoarthritis Progression and Treatment" was published in 2021. Journal: Comput Math Methods Med.

## Figures and Tables

**Figure 1:** Heat map of DEGs in the GSE72575 data set. Red represents upregulation of DEGs, and blue represents downregulation of DEGs. The expression intensity value comes from the gene expression levels analyzed by R software.

**Figure 2:** The enrichment analysis of GO function and KEGG signaling pathway of DEGs. (a) GO analysis. Blue represents MF (molecular function); gray represents CC (cellular component); orange represents BP (biological process). (b) KEGG enrichment analysis.

**Figure 3:** GSEA. The results showed that (a) ECM receptor interaction, (b) complement and coagulation cascades, (c) proteasome, (d) spliceosome, (e) focal adhesion, and (f) Nod-like receptor signaling pathway were significantly enriched in GlcN-treated MH7A cells.

**Figure 4:** PPI network diagram of DEGs. The nodes represent proteins, and the edges represent the interaction among these proteins.

**Figure 5:** Expression analysis of hub genes (a) IL6 and (b) DDIT3 in the GSE72575 data set.

## Data Availability

The data sets used and/or analyzed during the current study are available from the corresponding author on reasonable request.
